RETRACTED

# Exosomes derived from human umbilical cord mesenchymal stem cells promote osteogenesis through the AKT signaling pathway in postmenopausal osteoporosis

**DOI:** 10.18632/aging.204453

**Published:** 2022-12-27

**Authors:** Shi-Wei Ren, Guang-Qing Cao, Qing-Run Zhu, Min-Gang He, Fang Wu, Su-Mei Kong, Zhao-Yan Zhang, Qiang Wang, Feng Wang

**Affiliations:** 1 Department of Orthopedics, The Provincial Hospital Affiliated to Shandong First Medical University, Jinan 250014, Shandong, China; 2 Department of Spine Surgery, The Second Hospital, Cheeloo College of Medicine, Shandong University, Jinan 250033, Shandong, China; 3 Department of Gastrointestinal Surgery, Shandong Tumor Hospital and Institute, Shandong First Medical University and Shandong Academy of Medical Sciences, Jinan 250117, Shandong, China; 4 Department of Health, 960th Hospital of PLA, Jinan 250031, Shandong, China

**Keywords:** postmenopausal osteoporosis, exosomes, human umbilical cord mesenchymal stem cells, osteogenesis

## Abstract

Postmenopausal osteoporosis (PMO) is a relatively common disease characterized by low bone mass and microstructural changes of trabecular bone. The reduced bone strength is caused a variety of complications, including fragility fracture and sarcopenia. We used CCK-8 and EdU assays to evaluate cell proliferation rates. The osteogenesis effect was detected using ALP staining, alizarin red staining, and q-PCR. *In vivo*, the effects of exosomes derived from HUC-MSCs were evaluated using HE staining, IHC staining and Masson staining. In addition, we explored the mechanism of exosomes and found that the AKT signaling pathway played an important role in osteogenesis and cell proliferation. This paper mainly explored the function of exosomes derived from human umbilical cord mesenchymal stem cells (HUC-MSCs) and provided a new strategy for the treatment of postmenopausal osteoporosis. In conclusion, exogenous administration of exosomes can contribute to the treatment postmenopausal osteoporosis to a certain extent.

## INTRODUCTION

With the development of society and technology, human life is increasingly extending in length, and most women’s ages at menopause are approximately 45 to 55 years [1]. For a long time after menopause, the risks of various diseases increase. Postmenopausal osteoporosis (PMO) is a common disease in middle-aged and old women, mainly due to the lack of estrogen, which decreases the content of bone and promotes bone structural changes [2]. This can lead to an increased risk of fractures, which can lead to pain, complications, decreased quality of life and even death, causing burdens on families and society [3]. However, the underlying mechanism has not been fully explored. As previously reported [4, 5], osteoblasts and osteoclasts, which participate in bone formation and bone resorption, respectively, are important for bone homeostasis during bone remodeling. In addition, most of the existing treatments such as bisphosphate are very expensive and have many side effects, such as a cases have been reported that bisphosphonates can cause necrosis of the jaw bone [6], can also impair renal function [7].

RETRACTED

Recently, studies reported that exosomes derived from stem cells show great potential in tissue regeneration [8, 9]. Exosomes are extracellular vesicles with diameters of approximately 40–100 nm. Exosomes are released from a number of tissues and cells, mediating intercellular communication and transferring bioactive molecules, including DNA, microRNA, protein and lipids [10]. Compared with stem cells from other sources, human umbilical cord mesenchymal stem cells have the advantages of low immunogenicity, non-invasive harvesting procedures, easy *in vitro* amplification and ethical approaches [11]. There were three communication modes between osteoblasts and osteoclasts: direct contact, paracrine pathway and growth factor deposition in bone matrix. Exosomes from mineralized osteoblasts as well as osteoclasts and osteoblasts can participate in bone remodeling by promoting osteogenesis or osteoclast formation [12]. As previously reported, miR-214 contained in osteoclast-derived exosomes promoted osteoclast production by macrophages in bone marrow stromal cells via the PI3K/AKT pathway; thus, miR-214 contained in osteoclast exosomes caused pathological destructive bone disease [12]. Exosomes derived from osteoclast precursors activate osteoblast differentiation [13], while exosomes derived from osteoclasts inhibit osteoblast formation [14]. Therefore, exosomes play a major role in interventions for various diseases. Exosomes provide a potential, attractive and novel treatment for postmenopausal osteoporosis.

The phosphatidylinositol 3-kinase (PI3K) protein family is involved in the regulation of cell proliferation, differentiation, apoptosis and glucose transport [15, 16]. The PI3K/AKT pathway transmits signals from a wide-range of upstream regulatory proteins such as PTEN, PI3K and RTKs, and to many downstream effectors such as GSK-3β, FOXO, and MDM2, which are under control of various compensatory signaling pathways as well [17]. Activated AKT regulates cell functions by phosphorylating downstream factors such as enzymes, kinases and transcription factors. In this paper, we explored the function and mechanism of exosomes derived from human umbilical cord mesenchymal stem cells (HUC-MSCs), found that they played an important role in promoting osteogenesis and found that the AKT signaling pathway played an important role in osteogenesis and cell proliferation. Exosomes derived from HUC-MSCs has been often used in regenerative medicine and in the treatment of various diseases [11]. This paper provided a new strategy for the treatment of postmenopausal osteoporosis by using exosomes derived from HUC-MSCs.

RETRACTED

## MATERIALS AND METHODS

### Animal model and experiments

All animal procedures and experiments were provided by the Animal Laboratory of the Provincial Hospital affiliated with Shandong University. Animal experiments were conducted in accordance with the International Guidelines for Animal Research provided by the Council of International Medical Organizations (CIOMS) and approved by the Animal Ethics and Welfare Committee of the Shandong Provincial Hospital. Twenty-four 8-week-old female C57BL/6 mice (20±2 g) were housed under 12 h light/dark conditions, and food and water were offered ad libitum. The PMO model was established as previously reported [18]. The mice were placed in the prone position, chloral hydrate (Acmec, Shanghai, China, C11360) was used for anesthesia, hair was removed, skin was disinfected, a midline dorsal skin incision was made, the ovaries were removed with scissors, and the enterocoelia were sutured in turn until the skin. The sham group underwent a midline incision, removal the adipose tissue around the ovaries, and closure of the incision. Antibiotics (Cefuroxime sodium Zhijun, Shenzhen, China 0.5g/mouse) were given to prevent and treat infection after surgery, and the incisions were disinfected every day. Twenty-four mice (n=6/group) with PMO were randomly divided into four treatment groups: (1) PMO+PBS (Gibco, NY, USA C2001500BT) group; (2) PMO+Exos group; (3) PMO+bpV(phen) (Abcam, Cambridge, Britain, ab14436) group; and (4) PMO+Exos+MK-2206 (Beyotime, Shanghai, China, SF2712) group. (1) PMO+PBS (Gibco, NY, USA, C2001500BT) group: (1) PMO+PBS (Gibco, NY, USA, C2001500BT) group: Tail vein injection of PBS (Gibco, NY, USA, C2001500BT) 0.1 mL/mouse per day; (2) PMO+Exos group: Tail vein injection of exosomes derived from HUC-MSCs 100μg/mouse per day; (3) PMO+bpV(phen) Abcam, Cambridge, Britain, ab14436) group: Tail vein injection of bpV(phen) (Abcam, Cambridge, Britain, ab14436) 1μmol/mouse per day; (4) PMO+Exos+MK-2206 (Beyotime, Shanghai, China, SF2712) group: Tail vein injection of exosomes derived from HUC-MSCs 100μg and MK2206 (Beyotime, Shanghai, China, SF2712) 1μmol/mouse per day. The exosome was quantified by quantifying exosome proteins, the protein concentrations were measured using a BCA kit (Solarbio, Beijing, China, P0010). The treatments of these groups were established as previously reported [19–21]. All mice were treated for 8 weeks. All mice were sacrificed at 8 weeks. Bones of the lower extremities were collected for subsequent experiments.

RETRACTED

### BMCs isolation and culture from healthy and PMO mice

Cancellous bone was taken from the tibia and femur of experimental mice, periosteum and other soft tissues were stripped, and washed with sterile PBS (Gibco, NY, USA, C2001500BT) 3 times. In the DMEM (Gibco, NY, USA, C11995500BT) environment, cancellous bone was chopped to 0.5–1 mm^3^ size and then washed with PBS (Gibco, NY, USA, C2001500BT). Then, 0.25% trypsin (Gibco, NY, USA, 25200072) was added and digested in a 37° C constant temperature box for 20 minutes. 2 mL Fetal bovine serum (Gibco, NY, USA, 10099141) was terminated by digestion, and 5 times the volume of the red blood cell lysates (Solarbio, Beijing, China, R1010) were added. The lysates were centrifuged at 500 *g* for 5min, and the supernatants were removed. We added 1% collagenase type 1 (Gibco, NY, USA, 17100017), 37° C water bath to digest 1 h, 1000 r/min 5 min of centrifugation of the supernatants, and pellets were re-suspended in DMEM (Gibco, NY, USA, C11995500BT). We used 200 stainless steel mesh to filter and count cells. We made cell suspensions of 5×10^4^/ mL, injected into sterile petri dishes, cultured in 5% CO_2_ and 95% O_2_ in the incubator at 37° C, and changed the culture medium every 48 h. When cells were close to confluence, 0.25% trypsin (Gibco, NY, USA, 25200072) was used to pass the cells.

### Extraction and identification of exosomes derived from HUC-MSCs

A 10cm umbilical cord was taken from a sterile operating table, drained the blood and rinsed the surface blood with sterile saline. Put it into a 50 mL centrifuge tube containing 25 mL sterile PBS (Gibco, NY, USA, C2001500BT), and transfer them to a sterile operating table with a 4° C ice box. We carefully removed the umbilical artery and vein using scissors and forceps, Wharton’s Jelly was separated, and residual blood was washed with sterile PBS (Gibco, NY, USA, C2001500BT). Wharton’s Jelly was chopped to 0.5-1 mm^3^ size and then washed with PBS (Gibco, NY, USA, C2001500BT). The methods of digestion, isolation and culture were consistent with the extraction of BMSCs described above. HUC-MSCs were cultured for exosome extraction as previously reported [11]. Exosomes in FBS (Gibco, NY, USA, 10099141) were removed by Ultracentrifuge. Exo-free FBS (Gibco, NY, USA, 10099141) was used for HUC-MSC culture. The culture supernatant of HUC-MSCs from 3 to 6 generations was collected and used Ultracentrifuge (ThermoFisher Scientific, NY, USA, MTX/MX150) to centrifuge at 300 × *g* at 4° C for 10 min. Then, removed the precipitate in the centrifuge tube, the supernatant was centrifuged at 2000 × *g* for 30 min again, then collected supernatant was centrifuged at 10000 × *g* for 30 min, and supernatant was centrifuged at 140000 × *g* for 90 min again. The supernatants were removed, washed and precipitated with PBS (Gibco, NY, USA, C2001500BT), centrifuged again for 90 min at 140000 × *g*, the supernatants were removed, resuspended in 100 μL PBS (Gibco, NY, USA, C2001500BT), and frozen at -80° C until use. The morphology of exosomes derived from HUC-MSCs was observed using transmission electron microscopy (TEM) (JEOL, Tokyo, Japan, JEOL-1400 Flash) as previously reported [13]. The size distribution was analyzed using dynamic light scattering (DLS) (Malvern, London, Britain, Mastersizer 3000). The methods of exosomes proteins western blotting assay were consistent with the description of bone tissues or cells proteins western blotting assay in the following. Specific exosome biomarkers, including Calnexin (Abcam, Cambridge, Britain, ab265603), Alixs (Abcam, Cambridge, Britain, ab275377 1:1000), CD9(Abcam, Cambridge, Britain, ab236630 1:1000) and CD63(Abcam, Cambridge, Britain, ab134045 1:1000), were measured using western blotting assay, and according to the manufacturer’s instructions, the primary antibodies were diluted by primary antibody dilutions (Solarbio, Beijing, China, A1810).

RETRACTED

### Exosome labeling with PKH-26

PKH-26 red membrane dye (Solarbio, Beijing, China, D0030) was used for exosome labeling. 40 μL of PKH-26 (Solarbio, Beijing, China, D0030) and 500 μL of dilution buffer (Solarbio, Beijing, China, D0030) were mixed for exosome labeling. The prepared exosomes were cocultured with the mixture in the dark for 30 min. Then, 10% Exo-free FBS (Gibco, NY, USA, 10099141) was used to stop the staining reaction. The labeled exosomes were extracted at 100,000 × *g* for 1 h at 4° C with ultracentrifugation (ThermoFisher Scientific, NY, USA, MTX/MX150). The supernatant was removed, and the labeled exosomes were resuspended in 100 μL PBS (Gibco, NY, USA, C2001500BT) and cocultured with BMSCs for 24 h.

### 5-Ethynyl-2’-deoxyuridine (EdU) staining assay

DNA replication activity was evaluated by an EdU Apollo567 *in vitro* assay kit (Ribobio, Guangzhou, China, C10310-1) according to the manufacturer’s instructions to further determine the proliferation rate of cells. We made BMSCs cell suspensions of 5×10^4^/mL, injected into 96-well plate, cultured in 5% CO_2_ and 95% O_2_ in the incubator at 37° C, divided into three treatment groups: (1) Control group; (2) PMO+bpV(phen) (Abcam, Cambridge, Britain, ab14436) group and (3) PMO+Exos+MK-2206 (Beyotime, Shanghai, China, SF2712) group, with three replicates in each group. The logarithmic phase cells were cultured to the growth stage. According to the experimental specifications, the cells were cultured in medium at a 1000:1 ratio of dilution EdU (Ribobio, Guangzhou, China, C10310-1) solution for 4 h. Paraformaldehyde (Servicebio, Beijing, China, G1101) was used to fix cells for 20 min. Then, 0.1% Triton X-100 (Solarbio, Beijing, China, T8200) was used for permeation for 5 min. After staining with DAPI (Solarbio, Beijing, China, C0060), a confocal fluorescence microscope (ThermoFisher Scientific, NY, USA, DXRxi) was used for imaging.

RETRACTED

### CCK-8 assay

Cell proliferation was detected using the CCK-8 (Solarbio, Beijing, China, CA1210) assay. According to the manufacturer’s instructions, we made BMSCs cell suspensions of 5×10^4^/mL, injected into 96-well plate, cultured in 5% CO_2_ and 95% O_2_ in the incubator at 37° C. Divided into four treatment groups: (1) Control group; (2) PMO group; (3) PMO+Exos group; and (4) Exos Group, with three replicates in each group. The quantity of exosome added to BMSCs for the treatments was consistent with previous reports [19]. Control Group and PMO Group were added with Exo-free a-MEM medium (Gibco, NY, USA, C12571500BT), PMO+Exos Group (PMO BMCs treated with exosomes) and Exos Group (normal BMCs treated with exosomes) were added with 100μg/ mL exosome a-MEM medium (Gibco, NY, USA, C12571500BT). All groups were replaced with new a-MEM medium (Gibco, NY, USA, C12571500BT) as them required. The cell plate was cultured in the incubator, and 10 μL of CCK-8 (Solarbio, Beijing, China, CA1210) solution was added into each well and incubated in the incubator for 4 hours at 0 h, 24 h, 48 h and 72 h. An enzyme standard instrument (ThermoFisher Scientific, NY, USA, Multiskan SkyHigh) was used to measure the absorbance at 450 nm.

### Western blotting assay

The bone tissues or cells were digested in RIPA (Solarbio, Beijing, China, R0010) lysate containing protease/phosphatase inhibitor (Solarbio, Beijing, China, P1261) and PMSF (Solarbio, Beijing, China, R0010) and centrifuged at 13800 x *g* for 10 minutes at 4° C. The supernatants were removed, the protein concentrations were measured using a BCA kit (Solarbio, Beijing, China, P0010), loading buffer was added, and equal amounts of 20μg protein were electrophoresed using 10% SDS-PAGE (Solarbio, Beijing, China, A1010). The samples were concentrated at 80 V for 30 min and separated at 120 V for 1 h. The proteins were transferred to PVDF membranes (Millipore, MA, USA, ISEQ00010) at a constant current of 200 mA for 1 h. The membranes were blocked with 5%BSA (Solarbio, Beijing, China, SW3015) for 3 h, and according to the manufacturer’s instructions, the primary antibodies were dilutubted by primary antibody dilutions (Solarbio, Beijing, China, A1810). the primary antibody total-AKT (Abcam, Cambridge, Britain, ab8805 1:1000). p-AKT Thr308(Abcam, Cambridge, Britain, ab38449 1:1000), p-AKT Ser473 (Abcam, Cambridge, Britain, ab126433 1:1000), GAPDH Abcam, Cambridge, Britain, ab8245 1:1000) was used for incubation overnight at 4° C. After rinsing with TBST (Solarbio, Beijing, China, T1081), the secondary antibody (Solarbio, Beijing, China, SE134 1:5000) by 5%BSA (Solarbio, Beijing, China, SW3015) was incubated at room temperature for 1 h. After washing three times, the chemiluminescent signal was developed using ECL kit (Millipore, MA, USA, WBKIS0100) reagents in the chemiluminescent signal instrument (GE, USA).

RETRACTED

### Alizarin red staining assay

We made BMSCs cell suspensions of 5×10^4^/ mL, injected into 6-well plate, cultured in 5% CO_2_ and 95% O_2_ in the incubator at 37° C for 24 hours. Divided into four treatment groups: (1) Control group; (2) PMO group; (3) PMO+Exos group; and (4) Exos Group, with three replicates in each group. BMSCs with different interventions were cultured in six-well plates containing osteogenic differentiation medium (DMEM (Gibco, NY, USA, C11995500BT), 10%FBS (Gibco, NY, USA, 10099141), 10^-7^mol/L dexamethasone (Solarbio, Beijing, China, D8040), 5×10^-5^mol/L Vitamin C(Solarbio, Beijing, China, A8100), 0.1mol/L β-Glycero phosphate disodium salt pentahydrate (Solarbio, Beijing, China, G8100)). Control Group and PMO Group were added with Exo-free osteogenic medium, PMO+Exos Group and Exos Group were added with 100μg/mL exosome osteogenic medium. The osteogenic differentiation medium was changed every 3 days for 27 days. After washing the cells with PBS (Gibco, NY, USA, C20012500BT), the cells were fixed in 4% paraformaldehyde (Solarbio, Beijing, China, G1101) for 30 min. After the fixation solution was aspirated, the cell samples were washed with PBS (Gibco, NY, USA, C20012500BT) twice, and alizarin red dye (Solarbio, Beijing, China, G1452) was added for 5 min of staining. After staining, the cells were washed with PBS (Gibco, NY, USA, C20012500BT) twice. Finally, images were observed under a confocal microscope (ThermoFisher Scientific, NY, USA, DXRxi), and Image J was used to analyze the results.

### ALP staining assay

We made BMSCs cell suspensions of 5×10^4^/mL, injected into 6-well plate, cultured in 5% CO_2_ and 95% O_2_ in the incubator at 37° C for 24 h. divided into three treatment groups: (1) Control group; (2) PMO+bpV(phen) (Abcam, Cambridge, Britain, ab14436) group and (3) PMO+Exos+MK-2206 (Beyotime, Shanghai, China, SF2712) group. BMSCs with different interventions were cultured in six-well plates containing osteogenic differentiation medium. The osteogenic differentiation medium was changed every 3 days for a week. After washing the cells with PBS (Gibco, NY, USA, C20012500BT), the cells were fixed in 4% paraformaldehyde (Solarbio, Beijing, China, G1101) for 30 min. ALP dye (Solarbio, Beijing, China, BC2140) was added for 15 min of staining. The cells were washed with PBS (Gibco, NY, USA, C20012500BT) and observed under a confocal microscope (ThermoFisher Scientific, NY, USA, DXRxi). Image J was used to analyze the results.

RETRACTED

### RNA extraction, reverse transcription and qPCR

According to the manufacturer’s instructions, total RNA was extracted from cancellous bone or cells using Trizol reagent (Solarbio, Beijing, China, R1100). The total RNA of each sample was reverse transcribed to cDNA using the Evo M-MLV RT Premix (Accurate Biology, Changsha, China, AG11706) for qPCR. The SYBR Green PCR master mix (Accurate Biology, Changsha, China, AG11701) was used to conduct qRT-PCR in the Bio-Rad IQ5 real-time PCR system. The results were standardized with respect to U6 or β-actin, and gene expression analysis was performed using a 2^-ΔΔCt^ approach. The primers for β-actin were designed and synthesized by BioSune Biological Co., Ltd. All the sequences of the primers used for real time PCR: BMP2-F (Accurate Biology, Changsha, China; 12156): 5’-TGACTGGATCGTGGCACCTC-3’; BMP2-R(Accurate Biology, Changsha, China, 12156): 5’-CAGAGTCTGCACTATGGCATGGTTA-3’; RUNX2-F(Accurate Biology, Changsha, China, 12393): 5’-AGGGAATAGAGGGGATGCATTAG-3’; RUNX2-R(Accurate Biology, Changsha, China, 12393):5’-AAGGGAGGACAGAGGGAAACA-3’; PI3KR1-F(Accurate Biology, Changsha, China, 18708):5’-CTACTGTAGCCAACAACAGCATGAA-3’; PI3KR1-R(Accurate Biology, Changsha, China,18708): 5’-AAGGTCCCATCAGCAGTGTCTC-3’; PI3KCA-F(Accurate Biology, Changsha, China, 18706): 5’-AGCAGGAGAAGAAGGATGAGACA-3’; PI3KCA-R(Accurate Biology, Changsha, China, 18706): 5’-GTTGGTGAGCAGGATTCAGAGG-3’; PTEN-F(Accurate Biology, Changsha, China, 19211): 5’-TCCCAGTCAGAGGCGCTATGTA-3’; PTEN-R(Accurate Biology, Changsha, China, 19211): 5’-CCTTTAGCTGGCAGACCACAAAC-3’.

### Statistical analysis

SPSS software was used to analyze the data. All values are expressed as the mean ± standard deviation. Differences of multiple groups were compared by one-way analysis of variance (Fisher’s least significant difference [LSD]). A p value <0.05 was considered statistically significant.

## RESULTS

### Identification of exosomes derived from HUC-MSCs

Exosomes derived from HUC-MSCs were extracted by ultracentrifugation and were identified. Transmission electron microscopy (TEM) observations of exosomes derived from HUC-MSCs revealed the presence of spherical vesicles that were either circular or typically cup-shaped (Figure 1A). The size of exosomes derived from HUC-MSCs was analyzed using DSL, and the overall size distribution was 70 to 130 nm, which was consistent with previous reports [10] (Figure 1B). In addition, we confirmed the presence of markers, including Calnexin, Alixs, CD9 and CD63, from exosomes derived from HUC-MSCs using western blotting (Figure 1C). Moreover, PKH26 fluorescently labeled exosomes were recorded in BMSCs. PKH26-labeled exosomes were observed in the cytoplasm (Figure 1D).

RETRACTED

**Figure 1:** (**A**) The size and morphology of exosomes derived from HUC-MSCs were determined using transmission electron microscopy (TEM). (**B**) The size distribution of exosomes derived from HUC-MSCs was scattered and identified using DLS. (**C**) The surface biomarkers Alixs, CD9 and CD63 were detected using western blot to identify exosomes derived from HUC-MSCs. (**D**) The exosomes derived from HUC-MSCs were labeled with PKH26.

### Effect of exosomes derived from HUC-MSCs on BMSC proliferation and osteogenesis

Normal BMSCs and BMSCs extracted from PMO mice were cocultured with exosomes derived from HUC-MSCs to explore the effect of exosomes. A CCK-8 assay was used to measure the proliferation rate of cells. The results showed that the proliferation rate of BMSCs extracted from PMO mice was reduced compared with that of the control group on Days 1, 2 and 3. Exosomes derived from HUC-MSCs promoted the proliferation rate of BMSCs extracted from PMO mice (Figure 2A, 2B). In addition, we explored the osteogenesis effect of exosomes, and an alizarin red staining assay was performed. The results showed that the osteogenesis of BMSCs extracted from PMO mice was reduced compared with that of the control group. Exosomes derived from HUC-MSCs significantly improved the osteogenesis of BMSCs extracted from PMO mice (Figure 2C, 2D). Additionally, osteogenic genes, including BMP2 and RunX2, were analyzed by qPCR. The results showed that the expression of BMP2 and RunX2 was inhibited in BMSCs extracted from the PMO mouse group, and exosomes reversed the effect of PMO to promote the expression of BMP2 and RunX2 (Figure 2E, 2F). (*p < 0.05, **p < 0.01, ***p < 0.001).

**Figure 2:** (**A**) CCK-8 was used to detect the proliferation rates of BMSCs extracted from PMO mice. (**B**) The CCK-8 results were calculated using SPSS software, and significant differences are labeled. (**C**) Alizarin red assay was performed to evaluate the effect of osteogenesis. (**D**) The results of alizarin red staining were calculated using ImageJ software. (**E**) qPCR was performed to detect the expression of BMP2. (**F**) qPCR was performed to detect the expression of RunX2.

RETRACTED

### Mechanism of exosomes derived from HUC-MSCs in PMOs

As we previously reported, the AKT signaling pathway showed important significance in the regulation of bone metabolism [22]. Therefore, we explored the expression of key genes in the AKT signaling pathway using qPCR. The results showed that the expression of PI3KCA and PI3KR1 was inhibited in BMSCs extracted from the PMO mouse group, and exosomes promoted the expression of these genes (Figure 3A, 3B). PTEN is an important gene in the AKT signaling pathway [16]. We also investigated the expression of PTEN *in vitro*. PTEN was upregulated in the PMO group, and exosomes inhibited the expression of PTEN (Figure 3C). In addition, we explored the expression of AKT; total AKT and two phosphorylation sites, Thr 308 and Ser 473, were detected. The results showed that p-AKT was down regulated in BMSCs extracted from the PMO mouse group, and exosomes promoted the phosphorylation of AKT (Figure 3D–3F). (*p < 0.05, **p < 0.01, ***p < 0.001).

**Figure 3:** The expression of PI3KCA (**A**), PI3KR1 (**B**) and PTEN (**C**) was measured using qPCR in the control group, PMO group, PMO+Exos group and exosome group. (**D**) The expression of p-AKT (Thr308), p-AKT (Ser 473) and total-AKT were detected using western blotting in the control group, PMO group, PMO+Exos group and exosome group. The results of p-AKT (Thr308) (**E**), p-AKT (Ser 473) (**F**) were calculated using Image J software.

### Exosomes derived from HUC-MSCs promoted BMSC proliferation and osteogenesis through the AKT signaling pathway

We next verified the effect and mechanism of exosomes derived from HUC-MSCs. MK-2206, an inhibitor to inhibit the expression of AKT [22], and bpV(Phen) [15], a PTEN inhibitor, were used to investigate the mechanism of exosomes on cell proliferation and osteogenesis. The cell proliferation rate was detected by EdU staining. The logarithmic phase cells were cultured to the growth stage. The five groups of medium were replaced: Control group: Exo-free a-MEM medium; PMO group: EXO-free a-MEM medium; PMO+Exos group: 100μg/ml Exosomes and a-MEM medium; PMO+pbV(Phen) group: 1μmol/L pbV(Phen) and Exo-free a-MEM medium; PMO+ Exos +MK-2206: 100μg/ml Exosomes and 1μmol/L MK-2206 and a-MEM medium. Cocultured them for 24 hours under the same condition. The results showed that the positive EdU cells were promoted when cocultured with bpV(phen) in BMSCs extracted from PMO mice, and the positive EdU cells were inhibited when cocultured with MK-2206 in BMSCs extracted from PMO mice (Figure 4A, 4B). Osteogenesis was evaluated using ALP and alizarin red staining. The results showed that no significant difference was found between the control and PMO+bpV(phen) groups in ALP and alizarin red staining (Figure 4C–4F). When treated with MK-2206, the osteogenesis effect was significantly inhibited in the PMO+Exos group (Figure 4C–4F). The positive EdU cells, alizarin red and ALP area were evaluated using Image J software. (*p < 0.05, **p < 0.01, ***p < 0.001).

RETRACTED

**Figure 4:** (**A**) Cell proliferation was evaluated using EdU staining between the control group, PMO group, PMO+Exo group, PMO+bpV(phen) group and PMO+Exo+MK-2206. (**B**) The EdU-positive cells were calculated using ImageJ. (**C**) Alizarin red assay was performed to evaluate osteogenesis between different groups. (**D**) Quantitative calculation of alizarin red-positive areas. (**E**) We performed an ALP assay to evaluate osteogenesis between different groups. (**F**) Quantitative calculation of ALP-positive areas.

### Exosomes derived from HUC-MSCs promoted osteogenesis in PMO mice through the AKT signaling pathway

We verified the effect of exosomes derived from HUC-MSCs using a PMO mouse model. The results of HE staining showed that the bone tissue in the PMO group was significantly reduced compared with that of the control group. The exosomes derived from HUC-MSCs increased the bone volume, and the bone volume was significantly increased in the PMO+bpV(phen) group compared with the PMO group. MK-2206 significantly inhibited the effect caused by exosomes to reduce bone volume (Figure 5A, 5B). In addition, we performed Masson staining to evaluate the new bone formation rate. The results showed that new bone formation was significantly inhibited in the PMO group, and exosomes rescued this effect to promote new bone formation. Additionally, bpV(phen) inhibited PTEN to activate the AKT signaling pathway to promote new bone formation, and MK-2206 inhibited AKT expression to inhibit bone formation (Figure 5A, 5C). Moreover, we explored IHC staining to detect the expression of p-AKT. The results showed that the expression of p-AKT was inhibited in the PMO group, and exosomes promoted the expression of p-AKT when compared with the PMO group. In addition, bpV(phen) promoted the expression of p-AKT, and MK-2206 significantly inhibited the expression of p-AKT (Figure 5A, 5D). The positive areas of HE staining, Masson staining and IHC staining were evaluated using Image J software. (*p < 0.05, **p < 0.01, ***p < 0.001).

**Figure 5:** (**A**) HE staining, Masson staining and IHC (p-AKT) staining were performed to investigate osteogenesis between different groups. (**B**) The bone volume was calculated by HE staining using ImageJ. (**C**) The new bone formation rate was calculated by HE staining using ImageJ. (**D**) The expression of p-AKT was calculated by HE staining using ImageJ.

RETRACTED

## DISCUSSION

Postmenopausal osteoporosis is a problem faced by middle-aged and elderly women around the world and is characterized by bone fragility and skeletal deterioration [3, 23, 24]. A high risk of fragility fractures was the main complication in PMO patients [25], and the medical costs of fracture treatment has brought heavy economic burdens to society. Therefore, how to prevent and solve this problem has been studied by many academic researchers. Existing effective drug treatments, including denosumab and teriparatide, are costly [2]. Therefore, it is necessary to find new treatments that are cost-effective for PMO patients. In this experiment, exosomes derived from HUC-MSCs were used for PMO. Additionally, we investigated the mechanism of exosomes derived from HUC-MSCs to promote osteogenesis *in vitro* and *in vivo* through the AKT signaling pathway.

As previously reported, exosomes derived from mesenchymal stem cells showed potential in tissue regeneration [26, 27]. Zhang et al. [28] reported that exosomes derived from MSCs can promote osteochondral regeneration and that the effect of MSC-exosomes coordinated multiple cell types through regulation of the AKT signaling pathway and ERK signaling by AMPCP. Additionally, we previously reported that exosomes derived from MSCs can reduce apoptosis of osteocytes in glucocorticoid-induced osteonecrosis of the femoral head via the miR-21-PTEN-AKT signaling pathway [19]. All these findings indicated the potential of exosomes in skeletal regeneration. In this study, we extracted exosomes from the human umbilical cord, which is considered useless in obstetric operations. However, in our opinion, the advantages of umbilical cord mesenchymal stem cells were obvious, including easy access to sources, substantial presence of stem cells, and others. Therefore, we used HUC-MSCs for exosome extraction.

Additionally, we explored the effect of exosomes derived from HUC-MSCs. We mainly focused on the cell proliferation and osteogenesis effects. As we previously reported, exosomes derived from HUC-MSCs showed anti-apoptosis effects in glucocorticoid-induced osteonecrosis of the femoral head in rats [19]. Yang et al. [29] demonstrated that exosomes derived from human umbilical cord mesenchymal stem cells inhibited apoptosis through miR-1263 delivery to regulate the Hippo signaling pathway to prevent apoptosis in disuse osteoporosis. In this study, we explored the effect of exosomes derived from HUC-MSCs on cell proliferation and osteogenesis effects. We found that exosomes derived from HUC-MSCs can rescue the cell proliferation and osteogenesis of BMSCs extracted from PMO mice.

RETRACTED

The mechanisms of exosomes have been widely explored in previous studies [30–32]. Exosomal miRNAs accounted for more than 40% of RNA exosomes [33]. Therefore, previous studies reported that exosomal miRNAs play important roles in cellular functions, including apoptosis, cell migration and proliferation based on epigenetic modification [34–36]. In our study, we explored the mechanisms of exosomes at the protein level. As previously reported [16], PI3KCA promoted the phosphorylation of PI3K, thereby promoting the expression of osteogenic genes, while PTEN dephosphorylated PI3K and reduced its osteogenic effect. We found that exosomes derived from HUC-MSCs activated the AKT signaling pathway to regulate cell proliferation and osteogenesis. Additionally, we used a PTEN inhibitor and AKT inhibitor to lose and gain, respectively, the function of AKT signaling to explore the effect of exosomes. HE, Masson and IHC staining of the mouse model also verified the effect of AKT on osteogenesis.
